This article has been retracted.

# Analysis of Rotator Cuff Muscle Injury on the Drawing Side of the Recurve Bow: A Finite Element Method

**DOI:** 10.1155/2022/8572311

**Published:** 2022-08-16

**Authors:** Cheng Guo, Xinlong Liu, Yi Yang, Dong Zhang, Dan Yang, Jun Yin

**Affiliations:** ^1^Capital University of Physical Education and Sports, 100191 Beijing, China; ^2^Hebei Institute of Sports Science, 050011 Shijiazhuang Hebei, China; ^3^Beijing Sport University, 100084 Beijing, China; ^4^Tsinghua University, 100084 Beijing, China

## Abstract

**Background:**

This study establishes the shoulder model on the drawing side of recurve archers by the finite element method and finds out the stress changes on the rotator cuff muscles in the position of the humerus and scapula under different stages of special techniques. The aim of this study is to investigate the mechanism of rotator cuff damage on a recurve archer's drawing arm.

**Methods:**

A 22-year-old healthy male's shoulder CT and MRI data were collected, and the drawing side shoulder joint finite element model was constructed, which contains the structure of the shoulder blades, clavicle, humerus, supraspinatus, infraspinatus, teres minor, and subscapularis. The humerus on the drawing arm was simulated to raising the bow, drawing, holding, and releasing on the scapula plane, and stress changes in rotator cuff muscles are analyzed.

**Results:**

The peak stress on the infraspinatus increased slowly, and from the start of raising the bow to hold and release, the stress peak increased from 0.007 MPa to 0.009 MPa. The peak stress on teres minor rises slowly from 0.003 MPa at the start of raising the bow to 0.010 MPa at the moment of releasing. The peak stress in the subscapularis increased from 0.096 MPa to 0.163 MPa between the start of raising the bow and releasing. The peak stress on the supraspinatus varied greatly, and from the start of raising the bow to the start of drawing, the stress peak increased markedly from 1.159 MPa to 1.395 MPa. Subsequently, the stress peak immediately decreased to 1.257 MPa at the start of holding and then increased to 1.532 MPa at releasing.

**Conclusion:**

The position of the humerus and scapula would change with the different stages of special techniques. It causes stress changes in the rotator cuff muscles, and when the stress accumulates over time, the shoulder 5on the drawing side will gradually become injured and dysfunctional. In combination with the depth of the structural site and the surrounding structural features, corrective exercises can be used to prevent injury to the rotator cuff muscles.

## 1. Introduction

Recurve bow is a static sport that requires strength and endurance in the upper shoulder girdle of the torso. The body is characterized by asymmetries in applying force and the corresponding load. To take the arrow, the athlete must demonstrate a high focus standard while executing a sequence of repetitive, smooth, and consistently accelerated arm motions. One of the most prevalent injuries sustained by archers is a shoulder injury, which may be traced back to overuse, excessive load bearing, and the resulting friction, tugging, and extrusion of tissues between shoulders [1, 2]. Repeating significant movements necessitates the use of the drawing side shoulder.

There have included the supraspinatus, infraspinatus, subscapularis, and teres minor. The rotator cuff muscle is composed of these four muscles. Furthermore, maintain dynamic stability in the shoulder joint while also helping to perform active internal rotation, external rotation, and supination of the shoulder and providing a fulcrum for the other muscles of the shoulder [3, 4].

When abnormalities in the function of the rotator cuff muscles occur, they can lead to shoulder injuries. Most recurve archers suffer from rotator cuff injuries. The rotator cuff injuries are caused by inadequate musculature and muscular strength imbalances. Inadequate muscle strength can lead to compensations in the rotator cuff muscles in a centrifugal state [5]. For example, the supraspinatus is overused when it is used for prolonged periods to simultaneously abduct the shoulder and avoid superior humeral displacement [6, 7]. In addition, when there is an imbalance in the strength of the shoulder's internal and external rotator muscles, this can lead to tendonitis in the muscle [8, 9].

Elite recurve archers spend considerable time practicing real draws to develop their feeling of movement. Up to 1000 repetitions per day are required for training with the bow, including raising, drawing, holding, and releasing the bow. Due to the apparent repetitive nature of the bow arm shoulder's motion, the rotator cuff muscles become overworked, which leads to inflammation and injury [10]. Furthermore, minimal in-depth study shows that recurve archers suffer from rotator cuff muscle damage [11]. Long-term training may cause substantial damage to the rotator cuff muscles, affecting recurve archers' ability to carry out their daily routines [12].

A finite element approach seeks to break down large objects into tiny units with primary forms so that the pattern of parameters may be modeled in a simple manner [13, 14]. The 3D parameters of soft tissue could be acquired by combining CT and MRI scan data and enhancing the geometric similarity, boundary restrictions, and load similarity of the 3D finite element model. [15]. Finite element analysis has been employed by several research organizations [16–20].

Finite element analysis was used in this work after 3D reconstruction of the humerus, scapula, and rotator cuff muscles. Recurve bow contains four specific motions, and researchers wanted to see how the rotator cuff muscle was affected by tension during each action (Figure 1). We explore the origin of rotator cuff damage in recurve archers and offer a strategy for preventing injuries due to the absence, including in research of internal alterations in those other sports biomechanical testing.

## 2. Materials and Methods

### 2.1. Subject

The test subject was a healthy male club-level archer. He was 22 years old, 178 centimeters tall, and 90 kg heavy, with no prior injury or shoulder discomfort history, and the right side is the drawing arm, trained for 2 years.

### 2.2. Methods

CT and MRI scanning methods were used to capture pictures of the subject in a normal anatomical position, with the right arm in a relaxed state, vertical to the shoulder joint. The rotator cuff and bone were modeled 3D using CT and MRI data (Figure 2). CT and MRI pictures were limited to one millimeter in thickness.

The motion biomechanics of recurve archers were studied in the laboratory. For this study, eight infrared high-speed motion capture lenses from Sweden (Qualisys-OQUS700) were used to get the kinematic data that was needed (acquisition frequency: 200 Hz). The individual was instructed to put on a tight shirt and warm up during the test. Reflective markers were positioned at anatomical surface markers after the stretching. Sports biomechanics were able to record it and use it as the boundary condition for a finite element simulation of bow motion.

#### 2.2.1. Reconstruction of a 3D Model of the Drawing Arm's Shoulder Joint

For finite element analysis, Swanson Analysis, Houston, PA, USA, provided the application ANSYS19.1. Simulating a recurve bow's particular movement required the Static Structural module usage. Materialism's Mimics19.0 software (Leuven, Belgium) analyzed CT and MRI medical imaging data, resulting in a 3D reconstruction of the bone and the rotator cuff muscles. Bone and soft tissue were removed from each tomographic picture using software; also, a primary batch of 3D models was created in the opposite order. This was achieved by filling in the blanks on the surface of the 3D model, eliminating unwanted pixels, and smoothing out the edges to produce an almost-perfect geometric form and structure near the 3D model in terms of genuine human tissue. The scapula, clavicle, humerus, supraspinatus, infraspinatus, teres minor, and subscapular were all included in the final construction. Next, a finite element analysis program simulated the shoulder bone and muscle models in IGES format [22].

#### 2.2.2. Finite Element Model Reconstruction on the Drawing Side Shoulder

The biomechanical properties of the shoulder bone and muscles during the four significant recurve bow motions were examined in earlier investigations [23, 24]. The Static Structural module simulated the structural and mechanical stresses on the shoulder tissue.

The Static Structural module of the AnsysWorkbench19.1 program was used to import the existing 3D model shoulder bone and muscle files. The biomechanical test revealed the rotation angle of the humerus on the drawing arm, which was utilized to establish four separate movements. In the Ansys working interface, four linked simulation projects were formed. By studying the upper arm link's motion characteristics, it was possible to estimate the humeral angle for each of the four key times [25–27]. We utilized the findings of biomechanical 3D photography to establish the joint center positions of the elbow and shoulder when the bow was raising as the humerus assumed a common anatomical condition.

As part of our finite element simulation, we modelled the biomechanical changes in the structure of the shoulder tissue at four different stages of motion: raising, drawing, holding, and releasing. This was done to refer to previous research [28–30]. Meanwhile, for muscle and bone material qualities, isotropic linear elastic materials were used (Table 1).

#### 2.2.3. The Recurve Bow Characteristic Moment Simulation's Loading Mode

There were 1042 scapular and clavicle nodes secured and restrained in all. Two vectors were used to produce the plane ABC: AB in conventional anatomical position and AC at a regular time.

The shoulder coordinate's origin is the shoulder joint's A-center. The negative direction of the humeral vector AC would be used to create the shoulder *x*-axis. The shoulder coordinate system for finite element analysis uses a *y*-axis parallel to plane ABC's average vector. This identifies the humerus' rotation axis and direction.

The 720-node humerus model was selected. Biomechanical testing measured the humerus rotational load around the *y*-axis rotation angle in the created shoulder joint coordinate system. Two space vectors were constructed based on the four usual raising, drawing, holding, and releasing moments and the frame's shoulder joint and elbow point coordinates. The angle between the two space vectors was computed using formula (1). The angular stress of humeral rotation was then calculated using this information. The material parameters of the shoulder finite element model were determined according to previous study [21].

(1) $$\begin{array}{c} \text{available }\cos=\frac{\overset{⟶}{\text{AB}}∙\overset{⟶}{\text{AC}}}{\overset{⟶}{\left|\text{AB}\right|}∙\overset{⟶}{\left|\text{AC}\right|}}. \end{array}$$

## 3. Results

The infraspinatus' peak stress gradually increased. From drawing and holding the bow until releasing it, the peak stress rose from 0.007 MPa to 0.009 MPa. The peak stress in the teres minor rises slowly from 0.003 MPa at the start of raising the bow to 0.005 MPa at the start of holding. Following this, the peak stress increased to 0.010 MPa at the point of releasing. The peak stress in the subscapularis increased from 0.096 MPa to 0.150 MPa between raising and drawing; the peak stress then continued to grow to 0.161 MPa and 0.163 MPa at the start of holding and releasing. The supraspinatus peak stress rose from 1.159 MPa to 1.395 MPa between raising and drawing; it then fell to 1.257 MPa at the start of holding and climbed to 1.532 MPa at releasing (Table 2). Stress variations at each stage are indicated in Figures 3–18.

## 4. Discussion

The infraspinatus, teres minor, subscapularis, and supraspinatus muscles form the dynamic stability structure of the shoulder. The rotator cuff muscles encircle the shoulder capsule and the glenoid labrum. By contracting centripetally, the rotator cuff muscles enable the joint capsule to tighten. The supraspinatus and deltoid muscles keep the shoulder joint stable during an abduction. The subscapularis allows for internal rotation of the shoulder joint, while the infraspinatus and teres minor muscles help with the external process of the shoulder joint. They are all essential muscles that stabilize the shoulder joint [31]. Their stress changes directly affect the stability of the shoulder joint.

The peak stress in the infraspinatus muscle tends to rise gently except during the drawing to holding phase when the peak stress increases more rapidly. The stress rises quickly from the drawing stage to the holding stage. This variation reflects that the specific technique requires sustained force from the infraspinatus. When the infraspinatus muscle is weak, a muscle strength imbalance occurs with the internal rotators of the shoulder (pectoralis major, latissimus dorsi, rhomboid, etc.). The state of mechanical instability of the glenohumeral joint would lead to the shoulder injury.

During the first three stages of the particular technique of the recurve, the stress on the teres minor is lower. The stress on the teres minor increases suddenly at the stage of releasing. This indicates that the teres minor needs to be activated while exerting external rotation. This makes the muscle elasticity of the teres minor strongly influence the special techniques to recurve motion. When muscles are less flexible, this can lead to a higher risk of the teres minor injury [32].

The subscapularis muscle has the lowest stress value when raising the bowing stage. From the drawing stage, the subscapularis stress value increases and then remains at a constant level until the releasing. The specific technique of the recurve motion requires the drawing arm to be in prolonged abduction. The abduction movement causes the space below the rostral process to become narrow. The squeezed subscapularis puts stress on the tendon. This can lead to subscapularis injury [33].

The supraspinatus completes the supination of the humerus in the first three stages of the particular technique and presses down on the head of the humerus during the releasing stage. Frequent involvement of the supraspinatus in shoulder activities can put it under high tension for long periods. The supraspinatus is under increased stress for long periods, leading to muscle degeneration and injury [6]. The supraspinatus tendons can be damaged by impingement of the coracoacromial ligament and the acromion [34].

As a result, specific corrective exercises are required to enhance the force and prevent deformation and other problems. It improves muscle efficiency and prevents injury by reducing stress on the rotator cuff muscles, as well as helping to improve the performance of recurve archers.

## 5. Conclusions

After obtaining data from CT and MRI scans, a finite element model of the shoulder was developed, representing the in vivo glenohumeral physiological characteristic on the drawing side of the recurve archers [36].

Shoulder instability and injury can occur when the infraspinatus muscle strength decreases due to poor training. The sudden increase in stress of the teres minor at releasing indicates that it needs to be activated quickly. A decrease in muscle elasticity in the teres minor can lead to injury. The subscapularis is susceptible to compression and consequent damage due to the anatomy of the shoulder in which it is located. Supraspinatus is prone to acromioclavicular impingement and tendon degeneration.

The supraspinatus and subscapularis could be released to enhance the posture of the humeral head during abduction and the area beneath the acromion. This may help avoid muscle damage and dysfunction when combined with the depth and surroundings of the structural features. Corrective exercise can also enhance muscular strength, contributing to the recurve archer's improper and twisted shoulder action.

### 5.1. Limitation of the Study

The simulation results obtained in this research for the rotator cuff muscles are reliable to a certain extent, but further confirmation is needed with scientific cadaver studies.

## Figures and Tables

**Figure 1:** The four distinct movements of a recurve bow: start of raising, drawing, holding, and releasing (reproduced from Cheng et al. [21]).

**Figure 2:** Model establishment of the shoulder muscles and bones.

**Figure 3:** Stress changes at the start of the infraspinatus raising stage.

**Figure 4:** Stress changes at the start of the infraspinatus drawing stage.

**Figure 5:** Stress changes at the start of the infraspinatus holding stage.

**Figure 6:** Stress changes at the moment of the infraspinatus releasing stage.

**Figure 7:** Stress changes at the start of the teres minor raising stage.

**Figure 8:** Stress changes at the start of the teres minor drawing stage.

**Figure 9:** Stress changes at the start of the teres minor holding stage.

**Figure 10:** Stress changes at the moment of the teres minor releasing stage.

**Figure 11:** Stress changes at the start of the subscapularis raising stage.

**Figure 12:** Stress changes at the start of the subscapularis drawing stage.

**Figure 13:** Stress changes at the start of the subscapularis holding stage.

**Figure 14:** Stress changes at the moment of the subscapularis releasing stage.

**Figure 15:** Stress changes at the start of the supraspinatus raising stage.

**Figure 16:** Stress changes at the start of the supraspinatus drawing stage.

**Figure 17:** Stress changes at the start of the supraspinatus holding stage.

**Figure 18:** Stress changes at the moment of the supraspinatus releasing stage.

**Table 1:** The material parameters of the finite element model for the shoulder.

Materials	Elastic modulus (MPa)	Poisson's ratio
Muscle belly	1.08	0.49
Muscle tendon	1200	0.4
Bone	7300	0.3

**Table 2:** Stress peak of the rotator cuff muscles at each characteristic action of the recurve bow (MPa).

Muscle name	Raising the bow start	Drawing start	Holding start	Releasing
Infraspinatus	0.007	0.007	0.009	0.009
Teres minor	0.003	0.004	0.005	0.010
Subscapular	0.096	0.150	0.161	0.163
Supraspinous	1.159	1.395	1.257	1.532

## Data Availability

The data can be obtained through the responsible author.
